This article has been retracted.

# Application of Artificial Intelligence in Cardiovascular Imaging

**DOI:** 10.1155/2022/7988880

**Published:** 2022-01-12

**Authors:** Panjiang Ma, Qiang Li, Jianbin Li

**Affiliations:** The Affiliated People's Hospital of Ningbo University, Ningbo 315040, China

## Abstract

During the last two decades, as computer technology has matured and business scenarios have diversified, the scale of application of computer systems in various industries has continued to expand, resulting in a huge increase in industry data. As for the medical industry, huge unstructured data has been accumulated, so exploring how to use medical image data more effectively to efficiently complete diagnosis has an important practical impact. For a long time, China has been striving to promote the process of medical informatization, and the combination of big data and artificial intelligence and other advanced technologies in the medical field has become a hot industry and a new development trend. This paper focuses on cardiovascular diseases and uses relevant deep learning methods to realize automatic analysis and diagnosis of medical images and verify the feasibility of AI-assisted medical treatment. We have tried to achieve a complete diagnosis of cardiovascular medical imaging and localize the vulnerable lesion area. (1) We tested the classical object based on a convolutional neural network and experiment, explored the region segmentation algorithm, and showed its application scenarios in the field of medical imaging. (2) According to the data and task characteristics, we built a network model containing classification nodes and regression nodes. After the multitask joint drill, the effect of diagnosis and detection was also enhanced. In this paper, a weighted loss function mechanism is used to improve the imbalance of data between classes in medical image analysis, and the effect of the model is enhanced. (3) In the actual medical process, many medical images have the label information of high-level categories but lack the label information of low-level lesions. The proposed system exposes the possibility of lesion localization under weakly supervised conditions by taking cardiovascular imaging data to resolve these issues. Experimental results have verified that the proposed deep learning-enabled model has the capacity to resolve the aforementioned issues with minimum possible changes in the underlined infrastructure.

## 1. Introduction

With the widespread use of computers and the rapid development of related information industries, people have entered the age of informatization. The scale of application systems in various industries continues to expand, and the industry data generated is also exploding, just like a gold mine of data waiting for people to mine and use. At present, a large amount of unstructured image data has been reserved in the medical field, but the reuse rate of stored data still needs to be improved. Research statistics show that more than 80% of medical data comes from medical imaging, and more than 70% of clinical diagnosis requires medical imaging. Therefore, how to use medical imaging data more efficiently to improve diagnosis efficiency and medical level is a major challenge.

In recent years, the country is vigorously advancing the reform of medical information technology, and the application of cutting-edge technologies such as artificial intelligence to the field of medical diagnosis has become a new era choice. With the help of big data and AI technology, not only can the diagnosis efficiency and accuracy of diagnosis be improved and the diseases of countless patients be cured, but also they are helpful to improve the current situation of uneven distribution of medical resources in my country.

Nowadays, the number of deaths caused by cardiovascular diseases in our country is increasing year by year, and there is still a lack of effective cures. Relevant medical studies have shown that vulnerable plaques in the cardiovascular system are the main cause of a large number of cardiovascular diseases, and the current diagnosis of cardiovascular diseases mainly depends on doctors reading cardiovascular medical images. In addition, research statistics show that the amount of medical imaging data increases by about 40% every year, while the number of imaging doctors only grows by about 4.1%. Therefore, people urgently need a new technical means that can more efficiently automate the analysis of medical images to assist doctors in diagnosis and treatment. In recent years, artificial intelligence methods have emerged in an endless stream, and applications in various industries have also blossomed, especially in image-related fields, as shown in Figure 1, and the application of artificial intelligence and medical imaging. With the continuous enrichment of data sets and the growth of computing power, artificial intelligence has made significant progress in multiple visual tasks with high accuracy. The rate of target recognition and detection has become a reality. The hot development of artificial intelligence has caused a large number of scholars and researchers to enter this field, and the relevant technical details and theoretical foundations are constantly improving. And different from traditional machine learning that requires professionals to give specific rules before processing the image, artificial intelligence can learn the inherent effective features of the image by itself to improve the model effect, which will greatly alleviate the difficulties caused by the lack of doctors and experts in reality. Therefore, using artificial intelligence technology to solve the problem of automatic identification of diseased areas in cardiovascular medical imaging has become our first choice. At present, the diagnostic accuracy of artificial intelligence deep learning algorithms for some medical imaging lesions has exceeded the average level of doctors' diagnosis, and AI-assisted medical care is not out of reach. And there have always been related researches on automatically identifying the diseased area in medical images to improve the accuracy and reduce the time for experts to read the film. Even in 1995, there was the first auxiliary diagnosis system that used convolutional neural networks to automatically identify nodules in X-ray images [1]. In the past two years, neural networks have also shown a diagnostic level that surpasses doctors and experts in many medical image analysis fields, such as the use of brain CT images to detect intracranial microhemorrhage and DeepLung [2] network structure to detect lung nodules. Some time ago, Andrew Y.NG and others proposed CheXNet [3], which uses chest X images to detect pneumonia, which greatly encouraged the application research of deep learning in the field of medical image analysis.

In this paper, we have focused on cardiovascular diseases and use relevant deep learning methods to realize automatic analysis and diagnosis of medical images and verify the feasibility of AI-assisted medical treatment. The scientific contribution of this paper is given as follows:

- Deep learning-enabled approach is used to realize automatic analysis and diagnosis of medical images and verify the feasibility of AI-assisted medical treatment
- Weighted loss function mechanism is used to improve the imbalance of data between classes in medical image analysis, and the effect of the model is enhanced.
- The proposed system exposes the possibility of lesion localization under weakly supervised conditions by taking cardiovascular imaging data to resolve these issues
- To realize this achievement, we have tested the classical object based on a convolutional neural network and experiment, explored the region segmentation algorithm, and shown its application scenarios in the field of medical imaging

The rest of the paper is arranged according to the following agenda items.

In the subsequent sections, that is, in Sections 2 and 3, a detailed analysis of the existing state-of-the-art studies is presented, which is followed by the proposed model detailed description. Additionally, how the proposed model is formed and the working mechanism are explained in this section as well. In Section 4, experimental results are presented, and comparative analyses are reported. Finally, concluding remarks are given along with relevant references.

## 2. Related Work

Since the emergence of medical image scanning and computer storage technology, people have been working on an automatic image analysis system. A rule-based decision system has been developed since the 1970s, which extracts edge and line features through filtering and mathematical modeling and then analyzes images according to artificial rules. In the late 1990s, supervised learning methods began to emerge using training sets, training models using feature extraction, and statistical learning methods, leading to computer-aided diagnosis. Due to the limitation of manual feature extraction, a neural network model based on the hierarchical structure was developed and applied to medical image analysis in 1995 by LO [4].

Although neural networks developed well at the time, they did not attract much attention in their early days. Because of the limitations of computational power and the immaturity of theoretical research, early neural networks were difficult to train, and it was not until AlexNet [5] won the championship for ImageNet [6] in 2012 that AI deep learning algorithm came to the attention of the industry again. After years of research and development, deep learning technology has been widely used in the field of target detection. CascadedRCNN [7] structure improves the prediction by cascading multiple target detection networks based on different IOU thresholds to determine the training set of positive and negative samples and has achieved the best detection results on multiple public data sets. The Des [8] network structure successfully improves the semantic representation of shallow network features by introducing semantic segmentation surveillance information at a low level and then improves the detection effect of the model on small targets. Different from most target detection algorithms which detect the targets in images independently, Hu et al. [9] proposed a novel network structure that can improve the detection performance by learning the relationship between the targets. In addition, in order to solve the problem of loss of detail information caused by five downsampling processes in target detection and semantic segmentation network, the network framework of DetNet [10] reduces the downsampling process twice and introduces “Hole” convolution to increase the perception field of the model, and this provides an effective reference for the research of backbone network structure, which is especially suitable for detection and segmentation.

In the field of cardiovascular medical image analysis, the application of artificial intelligence-related technology has a long history. In 2017, a team from Stanford University used AI algorithms to analyze electrocardiograms and eventually outperformed the average of three experts in identifying them. Professor Xu's computer team developed a system in 2018 that artificial intelligence based on deep learning can be successfully used to identify coronary angiographic stenosis. Huo and Shan [11] analyzed the wide application prospect of supervised learning and unsupervised learning in artificial intelligence in cardiovascular disease diagnosis. Zeng et al. [12] completed the automated and accurate labeling of coronary CTA images; compared with the artificial method, it is more efficient and more complete. Christian Payer [13] proposed the ConvGRU depth network structure, which has reached the highest level in cardiac MRI case segmentation.

Due to the complexity of medical image analysis tasks and the lack of standard data, the multitask learning method has been widely used in medical image analysis. Based on the correlation between brain disease diagnosis and clinical score, Liu et al. [14] proposed a multitask, multichannel DM2L network structure. Clement et al. [15] improved U-Net, added a decoding branch, and completed Bright and Red classification in the field of fundus image, and the experimental results show that the multitask joint training method can achieve better results than the single-branch network. Qin et al. [16] proposed a network structure based on cardiac image sequences for simultaneous detection and segmentation of cardiac motion, and the experimental results show that the multitask training method is complementary to feature extraction. The Y-net proposed by Mehta et al. [17] contains both the diagnostic branch and the output branch, and the best results have been achieved in the medical imaging data set of breast tissue with a large reduction in the number of parameters.

In the field of medical image analysis, there are always some problems such as lack of accurate data or uncertainty labeling, so it is necessary to study the application of weak supervised learning in medical image analysis. With the rise of the deep learning technology of artificial intelligence, many tasks in image analysis, such as target delineation and focus location, require more information for labeling. Izadyyazdanabadi et al. [18] proposed a weak supervised learning method based on multiscale feature map fusion using training sets containing only hierarchical annotation information to complete the segmentation of regions of interest in CLE image data that is 88% more accurate than any other method in the same period. In order to solve the problem of fewer image data and more noise in real world, Navarro et al. [19] proposed a WSL network structure to solve the problem of more noise in network crawling image data, which provides a reference for introducing foreign data into the training process of neural network. The DEEPEM network model based on the EM algorithm is proposed by Zhu et al. [20]. It successfully borrows the weak monitoring data from EMRs and improves the result score of Luna 16 dataset by 1.5%.

Although deep learning has made great progress in the field of medical image analysis, the use of artificial intelligence in medical imaging diagnosis can also bring many benefits, such as improving diagnostic efficiency, improving diagnostic accuracy, and relieving medical resources, but there are still many problems. First, there is a lack of medical data with sufficiently refined labels. One is that medical data labeling needs to be done by professionals, and the other is that it is difficult to share at this stage. We all know that deep learning is a data-driven algorithm, and the lack of data is bound to impede the progress of medical AI. Secondly, the intelligent system using the deep learning model to complete the diagnosis is still lacking interpretability. Although the research on feature visualization of the deep learning model has been going on, it still has black-box characteristics in essence. Particularly in the field of medical diagnosis, the result of diagnosis is related to the physical and mental health of patients, so the interpretability of the model is very important.

## 3. Proposed Method

### 3.1. Medical Image Analysis Based on Artificial Intelligence

The specific execution process of using artificial intelligence to solve practical problems is very complicated, but its basic principle is very simple. First of all, a variety of sensors or manual inputs are used to collect a large amount of relevant data stored in the computer. Secondly, appropriate statistical learning or deep learning algorithms are used to model and analyze existing data according to specific problems. Finally, the computer calculates various possibilities in the real application scenario according to the collected current data and its own model and then outputs the decision with the highest probability. The process of using deep learning technology to solve the problem of medical image analysis is the same. The complete system consists of a basic layer, technical layer, and application layer. The base layer is mainly composed of physical devices for model calculation and data storage at the bottom layer. The technology layer uses various types of deep learning algorithms to build models and form effective core technologies. The application layer is the product and application formed by the combination of artificial intelligence technology and specific application scenarios.

As shown in Figure 2, the deep learning algorithm has achieved a level far superior to traditional image processing techniques in image classification, target detection, and semantic segmentation. Medical image analysis has become the main way of diagnosis of many serious diseases, but there are still many problems in the field of image diagnosis in China, such as a serious lack of experienced doctors, slow speed of image analysis, and high misdiagnosis rate. Medical images are taken by special imaging instruments, which are essentially image categories. Compared with general RGB images, medical image data standards are more unified, and there is no migration problem when applied to actual scenes. Therefore, it is of great practical significance to apply techniques such as image classification and target detection in the field of deep learning to solve problems such as disease diagnosis and lesion location in the field of medical images so as to improve diagnosis efficiency.

### 3.2. Deep Learning of Related Technical Foundation

#### 3.2.1. Basic Structure of Convolutional Neural Network

Compared with ordinary feedforward neural network, a convolutional neural network (CNN) has obvious advantages in image processing. Taking the AlexNet network structure as an example, CNN mainly contains structures such as convolution layer, maximum pooling layer, full connection layer, and nonlinear activation mapping, among which the convolution structure is the key structure of a convolutional neural network with strong feature extraction ability for images. The convolution operation process is shown in Figure 3.

In the figure above, the convolution kernel with the size of 2 × 2 slides on the feature graph with the step size of 2 completes the multiplication and summation operation of corresponding positions and then obtains the feature graph of the next layer. Compared with the fully connected layer, the convolution operation greatly reduces the number of network model parameters and thus reduces the risk of overfitting through the local perception and weight sharing operation.

Nonlinear activation mapping introduces nonlinear factors into the multilayer neural network and enhances the ability to fit the expression of the model. In general, the activation function needs to have the following properties: nonlinearity, monotonicity, and differentiability. The nonlinear property makes the neural network more expressive and can fit any nonlinear function. Monotonicity guarantees that a single layer network is convex. Differentiability ensures the normal operation of gradient backpropagation during model optimization. Commonly used activation functions include sigmoid and ReLU, defined as shown in (1) and (2). Compared with the sigmoid function, the ReLU function has the advantages of easy calculation and fast convergence, so it is used in the experiment.

(1) $$\begin{array}{c} \text{sigmoid}\left(x\right)=\frac{1}{1+e^{-x}}, \end{array}$$

(2) $$\begin{array}{c} \text{relu}\left(x\right)=\max\left(0,x\right). \end{array}$$

#### 3.2.2. Transfer Learning in Neural Networks

The deep neural network model contains a large number of parameters. If the data is not sufficient, it is easy to lead to the problem of overfitting. However, in practical application scenarios, it is difficult to have enough data to train a deep neural network model from the initial state. Therefore, it is necessary to apply the idea of transfer learning to the field of deep learning. Specifically, we usually use the classical large data set ImageNet to get initialization parameters through pretraining and then apply them to the new data set training. After fewer parameter updates, we get the network model suitable for the new data set. This training strategy is called neural network fine-tuning. The fine-tuning process is shown in Figure 4.

The application effect of neural network transfer learning is determined by many factors, the most important of which is the size of the new data set and the similarity of content features between the new data set and the source data set. Generally speaking, shallow layers of deep neural networks extract generic features, such as image texture, color, edges, and corners, and other basic image elements, which have certain universality for different data sets. However, higher-level networks are used to extract more abstract and global features, such as cat ears, dog ears, and other feature elements, which are generally only applicable to specific training data sets. Here are some of the main scenarios where we use transfer learning in deep learning:

1. The size of the new dataset is smaller than that of the source dataset, but the content of the two datasets is similar, which is the most common situation. Generally speaking, if the size of the new data set is too small, it may lead to an overfitting problem, which is not good for fine-tuning the deep convolutional neural network. Our general approach is to first use pretraining model parameters to initialize the network, then fix the shallow layer parameters, and learn the parameters of the high-level feature extractor and the output layer.
2. The new dataset has a large scale and some similarities with the source dataset in content. In this case, with a sufficient amount of data, we can try to update the entire network parameters with a small learning rate.
3. The new dataset is small in size and unrelated to the source dataset in content. In this scenario, the learning effect of transfer may not be obvious. Generally, we only update the parameters of the output layer to optimize the network so as to prevent the model from overfitting for a small amount of new data.
4. Compared with the original data set, the new data set is larger in scale but has great differences in content, such as migrating from the RGB image data set to the medical image grayscale. In this case, if the new data set is large enough, we can train a network model from scratch. However, it is found in practice that although the content of the image data set is irrelevant, training from loading the pretraining model is still more conducive to model convergence than random initialization. Therefore, we will use pretraining model parameter initialization to update the whole network model parameters normally according to loss changes.

Of course, the application of transfer learning in the neural network also has certain limitations. Because our new model parameters need to correspond to the source model parameters one by one, our new network model architecture needs to be consistent with the source model as well. For example, we cannot change the size of the convolution kernel and the number of basic network layers or arbitrarily change the number of characteristic channels and so on; otherwise, the value of migration parameters may be lost. In addition, due to the sharing of convolutional parameters, we can apply the convolutional network pretraining model to input images of different sizes. This is obvious in the case of only convolution and pooling layers, but it is still true in the case of fully connected (FC) layers with the help of 1 × 1 convolution operations because the fully connected layer and the convolution layer can be transformed into each other.

### 3.3. Weakly Supervised Learning

In real scenes, it is very difficult to obtain sufficient and accurate annotation data, and the deep learning model requires a large amount of data, so the ability of the deep learning model is often restricted by the size of the data set. In addition, some professional data sets need special personnel to collect and annotate, such as medical image data. In addition, due to the difference in professional level between different annotators, the labels provided may be inconsistent, which may lead to the failure of model training.

Generally speaking, weakly supervised learning is relative to fully supervised learning and unsupervised learning. Supervised learning is to train data with tags of high confidence that meet task requirements, such as classification task data with category labels, detection task data with category and coordinate box labels, and segmentation task data with pixel set category labels, so that the model can be fully fitted to complete the output task through training. Unsupervised learning means that the training data has no label, and the training data itself learns the inherent characteristics, such as clustering analysis and self-coding network learning. Weakly supervised learning refers to the situation where the acquired labels do not match the task requirements, or the label confidence is not enough, which can be divided into the following three categories:

1. Incomplete supervised learning: only a few parts of massive training data have labels, and a large number of samples do not have labels.
2. Inaccurate supervised learning: there is noise or even error in data labels.
3. Imprecise supervised learning: the granularity of data labels is too large, which does not meet the requirements of the task. For example, only image category labels are given in the target detection task.

In practical scenarios, medical images usually have category labels but lack lesions location labels. However, medical image annotation needs professional doctors and experts to complete, which leads to the high cost of large-scale data reannotation scheme. In the field of medical diagnosis, the interpretability of the model is particularly important, so automatic medical image analysis generally needs to complete the classification of lesions. Therefore, it is valuable to study the localization of lesions under uncertain supervision.

## 4. Experiments and Discussion

### 4.1. Experimental Data and Pretreatment

The experimental data of cardiovascular medical imaging in this study were all provided by a research institute of the Chinese Academy of Sciences. There are 1000 positive and negative samples each, and the image size is 350 × 7200. The positive sample image contains one or more lesion regions with uncertain size, while the negative sample image does not contain lesion regions. Each image has a corresponding category label, in which the positive sample lesion area label is the left and right abscissa value. In general, vulnerable plaques are characterized by fibrous cap thickness <65 *μ*m and lipid core area >30%. Our task consists of two parts: determining whether a given image is normal and detecting the abscissa range of the diseased portion. Different from general image analysis tasks, this topic has the following characteristics:

1. The experimental data in this paper are all single-channel grayscale images taken by medical imaging instruments, with relatively simple image content and lack of obvious structural features. However, commonly used basic network models such as AIexNet and VGG [21] are trained by RGB data sets such as ImageNet, so the initialization effect is not obvious by directly using pretraining model parameters.
2. There are only 2000 pieces of experimental data in this paper, and there is a high degree of similarity between images and a large amount of redundant information. Training a network model with high complexity will lead to overfitting problems.
3. Although the number of positive and negative samples in the experimental data is consistent, the area of the lesion area is much smaller than that of the normal area in the lesion area localization task, which also belongs to the quasi-imbalance problem, which easily leads to the bias of neural network learning and affects the judgment effect of the actual output.
4. The lesion region localization task needs to obtain the abscissa interval of the lesion region for each image, namely, [*X*_1_, *X*_2_], [*X*_3_, *X*_4_], and so on.

In fact, the lesion area division belongs to the category of semantic segmentation, but our label only has the abscissa range value without the pixel-level label. According to the characteristics of existing labels, we simplified the segmentation task into a regression task of label values of single-column pixels, which is equivalent to labeling 0, 1 for each column of pixels to indicate whether they belong to the lesion area. First, we need to change the coordinate range of the lesion area into a 720-dimensional 0, 1 label vector. Secondly, our image data is converted from the polar coordinates generated by the circular strafing of the imaging guidewire in the vascular cavity; that is, the most left end and the most right end of the image should be connected together. There is no full connection layer in our network structure, and the goal is to get a label vector with the same transverse length as the original image by regression output. Therefore, a certain area around the pixels of each column is needed to predict the label of the column.

From the analysis of the above sections, it can be seen that, due to the characteristics of image data, the classification network has less backpropagation information, and it is difficult to capture the characteristics of local lesions. The regression network can effectively achieve the classification of lesions but lacks the overall semantic information. Therefore, we expect to complete the integrated network model of image diagnosis and lesion region division, which not only meets the practical application requirements but also realizes the complementary advantages of multitask feature extraction capabilities. In fact, the idea of joint training has a long history, such as the classical target detection framework Faster RCNN [22] and YOLO series [23]. The network output contains both regional coordinates and regional categories. Moreover, experiments have proved that image features extracted by different training tasks are different, and the multitask joint training method can strengthen the feature extraction ability of the model and improve the detection and classification effect. The two-branch network model is mainly composed of three parts: shared convolutional layer, classification network branch, and regression network branch. Among them, the classification network branch also uses global average pooling (GAP) instead of the fully connected layer, which can not only effectively reduce the number of network parameters and get rid of the limitation on the size of network input but also help solve the problem of model interpretability. It should be noted that, different from the 2 × 2 pooling layer in the general network structure, according to the characteristics of the experimental image data and the network transmission requirements, we adopt a part of the 2 × 1 pooling structure.

As can be seen from Table 1, the superposition of 3 × 3 convolution kernels was used to replace 7 × 7 and 5 × 5 convolution kernels, and multiple nonlinear mappings were added [24] on the premise that the receptive field remained unchanged, enhancing the feature expression ability of the model. In the network model, classification network branches and regression network branches share the first several convolutional layers. In addition, we use the 1 × 1 convolution structure. The 1 × 1 convolution structure proposed by NIN [25] can realize the cross-channel fusion of information, increase the nonlinear expression ability of the network, and carry out dimension reduction or dimension enhancement in feature channel dimensions, which is widely used in various modern and advanced network models. In order to meet the demand of branch output of regression network, 1 × 1 convolution is used to achieve channel dimension reduction in this paper.

### 4.2. Experimental Design and Result Analysis

We divided the data set into 60% training set, 20% validation set, and 20% test set. Due to the high similarity between adjacent images, data may be collected from similar vascular regions, so it is important to randomly scramble the data before segmentation; otherwise, you may get high accuracy, which is actually not true. The initial learning rate was set at 0.001, and Adam optimizer [26] was used to train 70 epochs. The model parameters were saved when the loss value in the verification set was the lowest.

In the face of the problem caused by the imbalance of positive and negative samples, methods such as upsampling on a small number of samples or downsampling on a variety of samples are usually adopted, but they will have a great impact on the detection results, so the sampling method is not feasible. The method of changing the threshold value adjusts the classification output threshold parameter to make its value less than 0.5, even though the neural network has a greater possibility of identifying a certain area as a pathological area. The weighted loss method adjusts the weight of loss between positive and negative categories by lambda parameter. As shown in Formula (3), if we choose a relatively small lambda value, the output penalty when the ground truth is 0 [27] will be much smaller than when the ground-truth value is 1, so as to encourage the network to output non-0 even when the signal is weak. In practice, we can combine the two strategies and use the grid search method and validation set to find the best hyperparameter. In this paper, the evaluation of the detection effect includes the confidence level, and the change of threshold will affect the confidence level, so the weighted loss strategy is adopted. The branch loss function of the regression network is designed as follows:

(3) $$\begin{array}{c} {\text{Loss}}_{\text{regression}}=\left(y_{i}+\lambda \right)\frac{1}{n}\sum_{i=1}^{n}\left(-y_{i}\ln\;P_{i}-\left(1-y_{i}\right)\ln\left(1-P_{i}\right)\right). \end{array}$$

According to the test effect of the verification set, we selected the value of the hyperparameter lambda as 0. Lambda parameter value 0.5 does not change the average loss, but by observing the change of loss curve in the training process, we can see that the addition of class equalization mechanism can make the network converge better. The curve variation of the loss function is shown in Figure 5.

In this section, we conducted several groups of experiments and compared the improvement of the dual-branch combined training model in image diagnosis and lesion region classification with the AlexNet patch segmentation method as the benchmark. Meanwhile, the fppi-recall curve was separately drawn, which directly reflected the improvement effect of our model on recall rate under the premise of ensuring accuracy. As shown in Figure 6, in this section, we use the classical AlexNet and VGG classification network structure as the benchmark and use accuracy as the evaluation index to compare the results of the single-branch full-convolutional classification model and double-branch network classification results proposed by us. It can be seen that, with the increase of network depth and the number of parameters, VGG does achieve a better classification effect than AlexNet, but the increase is very limited. And for dichotomies, such accuracy is still very low. In order to be suitable for the dual-branch joint training model, we proposed a classification network containing 2 × 1 pooling layer. Although the number of parameters decreased a lot, the accuracy of using it alone also decreased. After the joint training, the classification accuracy greatly increased to 82.50%.

In conclusion, an increase of network depth in this experiment does not bring about a great improvement in the image diagnosis rate. As can be seen from the analysis in the preceding chapters, the main reason for the unsatisfactory classification effect is that the proportion of the lesion area used to distinguish the image is very small in the original image, and there is less backpropagation information. Although the simple increase of network depth can enhance the model learning ability, it also brings more network parameters. The dual-branch model greatly strengthens the constraints of the network on local information through regression network output and enables the shared convolution layer to better capture key features, thus greatly improving the classification effect. In addition, it can be seen from the experimental results that the weighted loss function strategy proposed by us improves the classification accuracy by about 5 percentage points, effectively alleviating the problems caused by the imbalance between classes.

As shown in Figure 7, patch segmentation and full convolution regression network were used as the benchmark in this experiment, and the score was used as the evaluation index of the effect of lesion region classification to compare the effect of our dual-branch network model. Score includes precision rate, recall rate, and regional overlap level. It can be seen that the classical patch segmentation method can effectively complete the task of lesion region division. We use a 30-pixel long slide window to slide horizontally in turn, and the output is processed according to the merge strategy described earlier. Patch segmentation is still a classification structure in essence, with a large number of repeated calculations and low efficiency. Therefore, we also compare regression networks based on full convolution. The regression network has a certain improvement in the effect, and the dual-branch structure greatly improves the effect of lesion region classification. Although some studies have shown that the classification network itself can capture spatial location information to a certain extent, the improvement of the effect of our model mainly comes from the effect of classification results on the final decision. Similarly, a weighted loss function strategy can greatly improve the effect of lesion region classification. Based on the above analysis, it can be found that class imbalance has a great impact on the learning of the network model. It should be noted that the weight hyperparameters determined by the verification set in this experiment are not necessarily the best choice, but the improvement effect is obvious, which also provides a reference for us to deal with similar problems in the future.

In the previous section, we compared the effects of different models by dividing scores into lesion areas. The score is a relatively scientific evaluation method, integrating three evaluation indexes: accuracy rate, recall rate, and regional overlap level. However, due to the particularity of the medical industry, we are more expected to obtain the highest recall rate on the premise of ensuring the accuracy rate, that is, to diagnose all disease variants as far as possible. Therefore, we separately evaluated the recall rate of lesion detection under different models and drew the recall-fppi curve as shown in Figure 8. It can be seen that, compared with the traditional patch segmentation method and the regression model of full convolution, the recall rate of our dual-branch joint training model is greatly improved, and the category balance strategy is also improved to some extent. In addition, on the whole, the dual-branch model with the weighted loss function strategy proposed by us also achieves the highest recall rate, which further proves the effectiveness of the scheme.

Our model is a dual-branch structure containing the output of classification results and regression results, which can carry out end-to-end learning and ultimately achieve the overall diagnosis of cardiovascular imaging and the function of lesion region division. Through multigroup comparative experiments, it is proved that the combined training method can greatly improve the effect of classification network and regression network without greatly increasing the number of parameters. In addition, the recall-coin PI curve can also prove that the dual-branch network model can obtain the highest recall rate on the premise of a high precision rate, which is in line with the actual demand. In addition, the use of the cross-modal pretraining model, stepwise training scheme, and weighted loss function strategy in the experimental process is of great help to the improvement of the model effect.

## 5. Conclusion

In recent years, the state has actively promoted the development of medical information, the application of advanced technologies such as big data and artificial intelligence in the medical field has become a trend and can not only save the lives of countless patients but also ease the strain of medical resources, and doctor-patient relationship is of great significance. In reality, a large number of disease diagnoses depend on medical imaging technology, so the content of automatic analysis of cardiovascular medical imaging based on deep learning conforms to the needs of the development of times and has important practical significance. In this paper, data and task characteristics of cardiovascular medical images are analyzed, and the edge region feature extraction is successfully solved by using image ring mosaic as preprocessing method. Next, we propose a joint training network with a classification branch and regression branch according to the task requirement. By sharing a convolution layer and using a regression network to extract local features, the diagnostic accuracy of the classification network is greatly improved, and the whole decision-making ability of the classification network is also improved. In addition, aiming at the problem of class imbalance in medical image analysis, we introduce the weighted loss function strategy, which improves the performance of the network and provides a reference for dealing with this kind of problem in the future. In addition, we have completed the experiment and research on the algorithm of cardiovascular focus localization under the condition of weak supervision. In real-world situations, there are not enough medical images with abundant labels, and the labeling of such data can only be done by doctors, so it is valuable to study the localization of lesions under weak supervision. Based on CAM theory, the single classification network completes the task of locating cardiovascular lesions and is helpful for the interpretability of the model. Although the accuracy is less than that under the condition of total supervision, it proves the significance of studying weak supervision learning. In addition, we introduce SE and SA modules to further improve the performance of CAM detection, and the performance of the basic network model is universal.

## Figures and Tables

**Figure 1:** Artificial intelligence and medical imaging.

**Figure 2:** Deep learning and medical imaging work model.

**Figure 3:** Convolution operation process.

**Figure 4:** Neural network fine-tuning process.

**Figure 5:** Comparison of loss curve changes during training.

**Figure 6:** Comparison of experimental results of different network structures.

**Figure 7:** Comparison of experimental results of different grid structures in lesion areas.

**Figure 8:** Multimodel recall-fppi result curve comparison chart.

**Table 1:** Double-branch network structure.

Layer name	Layer type	Classification branch	Regression branch
L1	Conv	(3 × 3,32) × 3(=7 × 7)	
		2 × 1 max pooling	
L2	Conv	(3 × 3,64) × 2(=5 × 5)	
		2 × 1 max pooling	
L3	Conv	(3 × 3,128) × 2(=5 × 5)	
		2 × 2 max pooling	2 × 1 max pooling
L4	Conv	(3 × 3,256)	(3 × 3,256)
		2 × 2 max pooling	2 × 1 max pooling
L5	Conv	(3 × 3,512)	(3 × 3,512)
		2 × 2 max pooling	2 × 1 max pooling
L6	Conv	(3 × 3,512)	(1 × 1,256)
		GAP	(1 × 1,1)
L7	Output	Output 1 (size 2 × 1)	Output 2 (size 720 × 1)

## Data Availability

The datasets used and analyzed during the current study are available from the corresponding author upon reasonable request.
